The article "A Study of Heat Shock Protein 90 and Serum CCL21 Expression in Pregnant Women with Preeclampsia" was retracted in 2023. Reasons: unreliable results or conclusions; concerns about the data; concerns about the peer review; concerns about the citations.

# A Study of Heat Shock Protein 90 and Serum CCL21 Expression in Pregnant Women with Preeclampsia

**DOI:** 10.1155/2022/1601431

**Published:** 2022-08-02

**Authors:** Weina Yang, Xuemei Yang, Su'e Zhang, Limei Zhang, Wenze Wang, Li Wang

**Affiliations:** Obstetrics Department, Shijiazhuang Obstetrics and Gynecology Hospital, Key Laboratory of Maternal and Fetal Medicine of Hebei Province, Shijiazhuang, Hebei, China

## Abstract

**Objective:**

The purpose of the study was to determine the significance of heat shock protein 90 (HSP 90) and serum chemokine ligand 21 (CCL-21) in pregnant women with preeclampsia (PE).

**Methods:**

From June 2021 to June 2022, the study enrolled 100 women undergoing obstetric examinations and delivering in our hospital; 50 PE patients undergoing routine obstetric examinations and delivering during the same period were enrolled in the research group; according to the severity, they were divided into mild PE and severe PE groups, while 50 healthy pregnant women undergoing obstetric examinations and delivering in our hospital during the same period were enrolled in the control group. In a subsequent analysis, serum levels of CCL-21 and HSP90 were compared between the two groups, and the correlation among CCL-21, HSP 90, and PE severity was analyzed.

**Results:**

An overall total of 50 patients with PE were enrolled in the study, which included 32 patients with mild PE and 18 patients with severe PE. Patients with severe PE had lower mean arterial pressure (MAP), HSP 90, and CCL21 index levels than those with mild PE; MAP, HSP 90, and CCL21 in the severe PE group were higher than those in the mild PE group, but the difference was not statistically significant; In the research group, MAP was weakly correlated with HSP90 concentration and CCL21 concentration, with correlation coefficients of 0.33 and 0.30, respectively, and the correlation analysis was significant.

**Conclusion:**

Patients with PE showed significantly increased serum concentrations of HSP90 and CCL-21, but a significant difference did not exist between mild and severe PE. In addition, there was a weak relationship between HSP90 and CCL-21 concentrations in PE patients and MAP, suggesting that HSP90 and CCL-21 play an instrumental role in the pathogenesis of PE, although more studies are needed to clarify the exact mechanisms.

## 1. Introduction

Preeclampsia (PE) is a common pregnancy-specific disease with potentially adverse outcomes for mothers and newborns, affecting approximately 3–5% of pregnant women [1]. Recent guidelines define PE as recurrent hypertension after 20 weeks of gestation with the following symptoms: urinary protein >300 mg/day; organ dysfunction (including renal insufficiency, liver dysfunction, and neurological or hematological complications); uterine complications including placental dysfunction (leading to fetal growth restriction). At present, anticoagulant drugs such as aspirin and low molecular weight heparin are widely used at home and abroad for the prevention of PE. The treatment of PE commonly relied on magnesium sulfate combined with labetalol and other antihypertensive drugs. Although effective in reducing the probability of its toxicity, the use of antihypertensive drugs during pregnancy poses certain risks to maternal and infant health [2]. Traditional Chinese medicine (TCM) classifies PE into the category of “sub-swollen” and “sub-halo” and believes that the location is mostly in the kidney and also in the liver and spleen and is attributable to qi stagnation and blood stasis. Medicines for calming the liver and suppressing wind, tonifying qi and strengthening the spleen, promoting blood circulation, and removing blood stasis are used for prevention and treatment. However, most TCM only evaluates the efficacy of the drug without clarifying its underlying mechanism of action.

Though great strides have been made in detecting and treating PE as early as possible, its prognosis still remains a significant issue in perinatal medicine [3]. As of now, little is known about the pathogenesis of PE, but it is closely associated with a number of factors, such as placental ischemia and vascular endothelial injury [4]. In the body, heat shock proteins (HSPs) are closely related to many cellular active factors, and they are important in the regulation of many physiological functions, such as cell proliferation, body development, and immunity; for example, when the body is under stress, heat shock proteins may be able to maintain cellular homeostasis [5, 6]. Heat shock protein 90, also called HSP90, is a protein that has been found to promote the folding and maturation of several client proteins through the ATP cycle with the participation of cochaperone proteins and then accurately control various biological processes such as gene expression, cell cycle, and proliferation [7]. Consequently, HSP90 is an important component of the cellular signal transduction network, which plays an important role in maintaining the homeostasis of the cellular environment. A chemokine can be defined as a class of small cytokines or signaling molecules secreted by cells that have the ability to stimulate chemotaxis in nearby cells. As a member of the CC chemokine subfamily, CCL21 is highly expressed in the T-cell region of high endothelial venules and lymph nodes of secondary lymphoid tissue in humans; there is an expression of its receptor CCR7 in naive T-cells, B cells, DC cells, and numerous tumor cells [8, 9]. In spite of their involvement in many functions of the body, HSP90 and CCL21 do not show any signs of expression during PE.

To investigate the mechanism of PE, this study included PE patients and compared the differences in their expression of HSP90 and CCL21 to the expression of these molecules in healthy pregnant women.

## 2. Materials and Methods

### 2.1. General Data

This paper is an exploratory study aimed at discovering the regularities and hypothesizing the related mechanisms. A total of 50 PE patients who underwent routine obstetric examinations and gave birth at our hospital between June 2021 and June 2022 were selected for the research group. Meanwhile, 50 healthy pregnant women with normal gestational age, pregnancy, and body mass index (BMI) were selected as the control group. Prior to the commencement of this study, all subjects signed an informed consent form voluntarily, and Shijiazhuang Obstetrics and Gynecology Hospital's Ethics Committee reviewed the consent form and approved it (No. 2019–22/254).

### 2.2. Inclusion and Exclusion Criteria

#### 2.2.1. Inclusion Criteria

All patients who met the following criteria were included in this study:

- Patients in the PE group who had been diagnosed with PE.
- Patients who had a singleton pregnancy.
- Patients whose results of HIV testing and other infectious diseases were negative.
- Patients who were aged less than 35 years of age.

#### 2.2.2. Exclusion Criteria

The following patients were excluded from the study:

- Patients had severe renal disease, gastrointestinal disease, coronary heart disease, mental illness, or alcoholism;
- Patients had recently experienced trauma or surgery (within one month);
- Patients previously had a cesarean section;
- Patients had no other health records except for those related to gestational diabetes mellitus.

### 2.3. The Diagnostic Criteria

The criteria for preeclampsia: the first occurrence of systolic blood pressure ≥140 mmHg or diastolic blood pressure ≥90 mmHg after 20 weeks of pregnancy, and proteinuria, that is, urine protein ≥0.3 g/24 h. At least one of the following criteria can be diagnosed as severe preeclampsia: two systolic blood pressure ≥160 mmHg or diastolic blood pressure ≥110 mmHg for patients on bed rest 6 hours apart; proteinuria: ≥5 g/24 h or twice urine protein at 4-hour interval; oliguria: 24-hour urine output <500 ml; brain or visual disturbances; pulmonary edema or cyanosis; epigastric or right upper quadrant pain; impaired liver function; platelets decreased; fetal growth restriction.

### 2.4. Observation Indicators

The patient's age, gestational age, parity, BMI, blood pressure, and other information were collected at the time of admission, fasting venous blood was collected in the morning upon admission, and enzyme-linked immunosorbent assay (ELISA) tests were used to determine the levels of HSP90 and CCL21 in peripheral blood. All ELISA kits were obtained by Thermo Fisher Scientific (US), with the cat no. BMS2090 of HSP90 and cat no. 88-58214-22 of CCL21.

### 2.5. Statistical Analysis

All data analysis were performed using SPSS 22.0, and graphs were visualized using *R* software. The measurements were expressed as (mean standard ± deviation), while the counts were expressed as a rate; a *t*-test and chi-square test were conducted to determine whether a statistical difference existed between the groups. Correlation analysis between measurement data was performed using individual correlation analysis. All outcomes were calculated at *α* = 0.05 as the limit of statistical significance.

## 3. Results

### 3.1. General Data Comparison

The results of Table 1 indicate that there was no significant difference between the control and PE groups in terms of general characteristics such as age, gestational age, parity, and body mass index. Compared to the control group, the PE group had elevated systolic and diastolic blood pressures, and the difference was statistically significant (all *P* < 0.05).

#### 3.1.1. Comparative Analysis of the Expression Levels of MAP, HSP 90, and CCL21 between the Two Groups of Patients

As can be seen in Table 2, the MAP, HSP 90, and CCL21 levels in the research group showed an upward trend as compared to the control group (all *P* < 0.05).

### 3.2. Comparison of MAP, HSP 90, and CCL21 Expression Levels among Patients with Different Stages of PE

Table 3 shows a higher level of MAP, HSP 90, and CCL21 in the patients with severe PE as compared to those with mild PE, but the differences were not statistically significant (all *P* > 0.05).

### 3.3. Analysis of Correlation between HSP90, CCL21, and MAP in the Research Group

MAP levels in the research group were weakly correlated with HSP90 and CCL21 concentrations, with correlation coefficients of 0.33 and 0.30, respectively (all *P* < 0.05) (Figure 1).

## 4. Discussion

It is believed that PE is one of the main causes of maternal mortality worldwide, and the perinatal mortality rate for PE-affected pregnant women is five times higher than for normal pregnant women [10]. Although the exact cause of PE has not been fully elucidated, it is associated with abnormalities of the placenta during the first trimester of pregnancy. Cytotrophoblast cells invade the uterine spiral arteries during normal pregnancy, causing the arterioles to dilate [11]. However, in PE, the cytotrophoblast cells are unable to adequately invade the spiral arteries, resulting in a decreased placental blood flow and increased placental oxidative stress [12]. Since the symptoms of PE are atypical in the early stages, the study of serum markers may help to explain the pathogenesis of PE at the level of proteins, as well as provide a means of detecting, monitoring, and preventing it.

The results of this study showed that MAP, HSP90, and CCL21 in PE patients were significantly higher than those in normal pregnant women; HSP90 and CCL21 in the severe PE group were higher than those in the mild PE group, but the difference was not statistically significant. Both HSP90 and CCL21 concentrations were weakly correlated, with correlation coefficients of 0.33 and 0.30, respectively. HSP is a highly conserved molecule and a major molecular regulator whose expression is enhanced by various stress conditions and is involved in protein homeostasis [13]. As one of the main HSP proteins, HSP90 is a vital node of the cell signal transduction network, which is vital to maintaining the homeostasis of the intracellular environment [14]. The HSP90 receptor protein has been identified as closely related to apoptosis and signal transduction. In response to stimuli from the outside world, HSP plays an important role in stimulating or reactivating cell death [15, 16]. There is evidence that HSP90 is highly expressed in placental trophoblast cells, and it is speculated that this increase may be the result of secondary mechanisms, such as inflammation, but is not necessarily the cause of the symptoms of PE [17]. Chemokines are multiple-function mediators which are primarily involved in the mobilization of leukocytes to inflammatory tissues [18]. In the progression of tumors, CCL21 plays a dual role, promoting the immune response to the tumors while causing metastasis of tumor cells into lymph nodes that are overexpressed with SLC [19]. The lack of significant results in this study may be related to the small sample size. The research on the relationship between CCL21 and eclampsia has not been reported up to now, but it can be speculated that CCL21 may play a role in the pathogenesis of eclampsia. The results of Coşkun Güzel et al. showed that HSP90 was significantly elevated in the third trimester and may play a role in the pathogenesis of preeclampsia [17].

However, this study has the following limitations. First of all, this study is not a randomized controlled study, and the reliability is low. Secondly, this study is a clinical study, only the concentration and correlation of HSP90 and CCL21 were discussed, and the mechanism between them was not studied in depth.

## 5. Conclusion

In conclusion, serum concentrations of HSP90 and CCL21 were significantly higher in PE patients, but there was no significant difference between mild and severe PE. In addition, the concentrations of HSP90 and CCL21 in PE patients were weakly correlated with MAP, which suggests that they are associated with the pathogenesis of preeclampsia, but the specific mechanism remains to be determined.

## Figures and Tables

**Figure 1:** Correlation analysis of the MAP concentration with the concentrations of HSP90 and CCL21.

**Table 1:** Comparison of general data of the two groups of patients.

	Control group (*n* = 50)	Research group (*n* = 50)	*t*/*x*^2^	*P*
Age (years)	28.61 ± 5.85	29.48 ± 6.22	0.72	0.47
Gestational week	35.12 ± 3.56	34.11 ± 4.25	1.29	0.20
Parity (primi/parity)	24/26	29/21	1.00	0.31
SBP (mmHg)	118.85 ± 18.59	149.58 ± 22.54	7.44	<0.001
DBP (mmHg)	72.59 ± 14.52	101.25 ± 23.33	7.38	<0.001
Body mass index (kg/m2)	30.24 ± 5.26	31.08 ± 5.11	0.81	0.42

**Table 2:** Comparison of the expression levels of MAP, HSP 90, and CCL21 in the two groups of patients.

	MAP	HSP 90	CCL21
Research group (*n* = 32)	128.59 ± 22.28	1.27 ± 0.34	139.86 ± 17.74
Control group (*n* = 18)	89.14 ± 13.47	0.92 ± 0.23	112.24 ± 13.47
*t*	10.71	6.03	8.77
*P*	<0.001	<0.001	<0.001

**Table 3:** Comparison of expression levels of MAP, HSP 90, and CCL21 in patients with different degrees of eclampsia.

	MAP	HSP 90	CCL21
Mild PE (*n* = 32)	121.63 ± 15.83	1.24 ± 0.31	136.21 ± 24.18
Severe PE (*n* = 18)	126.61 ± 10.93	1.41 ± 0.37	146.33 ± 26.70
*t*	1.183	1.725	1.368
*P*	0.243	0.089	0.178

## Data Availability

No data were used to support this study.
